This article has been retracted.

# Type 2 Diabetes Mellitus (T2DM) and Carbohydrate Metabolism in Relation to T2DM from Endocrinology, Neurophysiology, Molecular Biology, and Biochemistry Perspectives

**DOI:** 10.1155/2022/1708769

**Published:** 2022-08-09

**Authors:** Hilla Mills, Ronald Acquah, Nova Tang, Luke Cheung, Susanne Klenk, Ronald Glassen, Magali Pirson, Alain Albert, Duong Trinh Hoang, Thang Nguyen Van

**Affiliations:** ^1^Department of Medical Science, University for Development, Accra, Ghana; ^2^RD Lab, The Hospital Institute for Hebal Research, Toluca 50200, MEX, Mexico; ^3^Research Institution of Clinical Biomedicine, Hospital University Medical Centre, Ulm 89000, Germany; ^4^Industrial Research Group, International College of Science and Technology, Route de Lennik 800, CP 590, Brussels 1070, Belgium; ^5^Clinical Analysis Lab, Center of Bio-Medicine, Hanoi, Vietnam

## Abstract

Type 2 diabetes mellitus (T2DM) is a severe disease caused by metabolic disorders, particularly carbohydrate metabolism disorders. The disease is a fatal global trouble characterised by high prevalence rates, causing death, blindness, kidney failure, myocardial infarction, amputation of lower limps, and stroke. Biochemical metabolic pathways like glycolysis, gluconeogenesis, glycogenesis, and glycogenolysis are critical pathways that regulate blood glucose levels with the glucokinase (GK) enzyme playing a central role in glucose homeostasis. Any factor that perturbs the aforementioned biochemical pathways is detrimental. Endocrinological, neurophysiological, and molecular biological pathways that are linked to carbohydrate metabolism should be studied, grasped, and manipulated in order to alleviate T2DM global chaos. The challenge, howbeit, is that, since the body is an integration of systems that complement one another, studying one “isolated” system is not very useful. This paper serves to discuss endocrinology, neurophysiology, and molecular biology pathways that are involved in carbohydrate metabolism in relation to T2DM.

## 1. Introduction

According to Tramunt et al. [1], diabetes is more prevalent in men, especially in the middle-aged individuals, than in women. This is a general trend all over the world except some few parts like North Africa and the Middle East. The International Diabetes Federation's last global estimates in 2017 indicated that diabetes prevalence is larger in men than in women (9.1% vs. 8.4%, respectively). This information suggested that approximately 12.3 million more men lived with diabetes than women. The clinical and experimental evidence that support the discrepancies in diabetes prevalence are mainly based on sex hormones endocrinology. The postpubertal sex steroid hormones in particular account for different diabetes prevalence rates in men and women. Premature ovarian sufficiency and early menopause in women correlate with an increased risk of developing T2DM more than premenopausal ones. A documented reduction in diabetic menopausal women incidence of about 21–35% was due to an oestrogen-based hormonal therapy. Hypogonadism men are at risk of developing T2DM and vascular ailments. It is reported that testosterone supplements improve both glucose and lipid homeostasis. It is beyond dispute that the highlighted endocrinology triggers and influences other biological pathways like glucogenesis, glycolysis, and neuropathways that are associated with homeostasis, particularly glucose and lipid homeostasis. Besides, herbal medicine and nanomaterials have also been used in medical engineering [2, 3].

## 2. Challenges Associated with T2DM Studies

Gender, as highlighted above, is one of the challenges in treating T2DM. A thorough understanding of male and female physiology in relation to T2DM is imperative. Tramunt et al. [1] asserted that gender governs energy storage and use. Females can withstand undernutrition periods better than males, and this enables females to preserve their reproductive functions. Most importantly, gender determines carbohydrate and lipid metabolism. It is reported that females are more insulin sensitive than males. The list of differences goes on and on. This means glucose and lipid metabolism in men and women is not the same. Tramunt et al. [1] argued that there should be sex-specific medicine for T2DM. Achieving this goal is very expensive considering that research projects are done for men and women separately. This sounds to be the major drawback of the idea of sex-specific T2DM medicine. Notwithstanding, if the goal is achieved, a number of T2DM patients will lead almost a normal life.

Other daunting factors when it comes to T2DM treatment are age, race, health status, and so on. Focusing on health status, recent studies showed that angiotensin-converting enzyme 2 (ACE2) is a receptor of the severe acute respiratory syndrome corona virus (SARS-CoV). The ACE2 is overexpressed in diabetic and hypertension patients due to the use of angiotensin-converting enzyme 1 (ACE1) inhibitors. Consequently, patients suffering from T2DM and hypertension are at risk of acquiring the COVID-19 diseases, and once such patients get sick, death rates for this group are high. It is imperative to monitor glucose levels in SARS-CoV patients. Needless to say, the job is irksome [4]. Studying T2DM is complex considering factors that affect glucose homeostasis. Healthy T2DM animal models are of great help in studying the disease. However, in the world, comorbidity is a great challenge.

According to Timer et al. [5], T2DM affects many body systems like cardiovascular and nervous systems. A plethora of studies revealed that T2DM is a risk factor for vascular dementia and Alzheimer's disease. Studies that aimed to investigate the correlation between T2DM and cognitive impairment have been done, and they focused on the presence of apolipoprotein allele, mitochondrial malfunction, oxidative stress, macrovascular mechanisms, the formation of advanced glycosylation end-products, inflammation, and insulin resistance [6]. Patients who suffer from diabetic retinopathy showcased a poor cognitive skill compared with disease-free patients. The observation is attributed to microalbuminuria in T2DM patients. Timer et al. [5] conducted a study to compare T2DM-peripheral-neuropathy patients and T2DM-peripheral-neuropathy-free patients concerning cognitive functions based on the notion that peripheral neuropathy may also correlate with microvascular impairment in the brain. The team observed no significant differences between the TDM patient groups. Such investigations still need to be expanded since only a handful studies have been done. Howbeit, polyneuropathy manifests in the early phases of T2DM, and needless to say, T2DM interferes with the nervous system.

Feng et al. [6] designed an experiment to probe the relationship between TSH (thyroid-stimulating hormone) and serum uric acid (SUA) in T2DM patients with early-stage diabetic kidney disease (ESDKD). A negative correlation of 0.35 (95% confidence interval) between SUA and TSH was reported. This implies that T2DM patients with ESDKD whose SUA levels are high have decreased TSH levels. Uric acid (UA) is produced following purine metabolism. The kidney eliminates about 70% of UA. Recent studies reveal that SUA causes the development of microvascular diseases. According to De Cosmo et al. [8], SUA significantly correlates with albuminuria in T2DM patients. As a result, hyperuricemia has been used as a “biomarker” for DKD prediction. It is documented that thyroid dysfunction can exacerbate glucose metabolism and induce hyperglycaemia in T2DM patients, thus promoting the risk of diabetic complications. Hyperglycaemia lowers the level of thyroid-stimulating hormone (TSH) and mitigates the conversion of thyroxine to triiodothyronine in the peripheral tissues. This piece of evidence without doubt proves that there is a link between endocrinology and T2DM.

According to Stoll et al. [9], secretion of insulin is governed by a circular RNA that contains a lariat sequence of the second intron insulin gene. A decrease in the expression of key components of the secretory machinery of *β*-cells that leads to impaired glucose or KCl-induced insulin release and calcium signalling was reported following silencing of this intronic circular RNA in pancreatic islets. The effect of the circular RNA was observed to be exerted at the transcriptional level. It is reported that this effect involves an interaction with the RNA-binding protein TAR DNA-binding protein 43 kDa (TDP-43). The level of this circularised intron is mitigated in the islets of rodent diabetes models and of T2DM patients. This is possibly due their impaired secretory capacity. Type 2 diabetes mellitus, therefore, can be studied from a molecular biology perspective.

The xenobiochemistry concept of T2DM with respect to *ω*-6 PUFA-rich vegetable cooking oil we use almost daily to cook our meals at home is elucidated by Yamashima et al. [10]. Hydroxynonenal is a compound that forms following lipid peroxidation. It is also formed during vegetable oil deep-frying. The phenomenon is frequent when using soybean, rapeseed, and sunflower vegetable oil that contain a lot of linoleic acid. Reactive oxygen species attack membrane *ω*-6 PUFAs to generate endogenous hydroxynonenal. It is reported that hydroxynonenal forms adducts with 4 amino acids, namely, arginine, lysine, histidine, and cysteine. It is thought that the compound might be able to interfere with proteins. Therefore, hydroxynonenal is capable of causing neuron dysfunction and degeneration by altering membrane-associated glucose and glutamate transporters, ion-motive ATPases, enzymes involved in amyloid metabolism, and cytoskeletal proteins. Recently, hydroxynonenal is increasingly recognised as a particularly important mediator and marker of cellular dysfunction and degeneration in diverse disorders such as T2DM, arteriosclerosis, cardiovascular disease, and stroke.

This paper serves to shade some light on the critical neurophysiological, endocrinological, biochemical, and molecular biological aspects in relation to T2DM. It is imperative that the readers should bear in mind that the study assumes the only disease in *the test subjects* is T2DM. The major enzyme GK and its activities, the CNS and carbohydrate metabolism, and some mechanisms related to T2DM are discussed herein.

### 2.1. Carbohydrates

Simple sugars are either monosaccharides or disaccharides that are easy to break down resulting in a rapid increase of blood sugar. Consequently, a rapid secretion of insulin occurs. Examples of such sugars are ribose, fructose, galactose, maltose, glucose, lactose, and sucrose. Sources of such sugars are carbonated beverages, honey, table sugar, fruit juice, candy, and corn syrup [11].

There are sugars that are either disaccharides or polysaccharides having a complex chemical structure. These sugars are not easy to break down, and thus they do not cause a rapid blood sugar escalation following consumption. Sugars such as amylose, dextrin, cellulose, cellobiose, and rutinulose fall under complex sugars. The sugars are found in foods like apples, brown rice, unrefined whole grains, broccoli, spinach, and lentils. Thousands of glucose units are joined together within starches. The starches fall under complex sugars. Wheat, pasta, potatoes, and chickpeas are sources of starches [11].

Complex carbohydrates that are not digestible belong to this group of sugars. The sugars encourage bacterial growth in the colon. As a result, defecation is made easy. It is reported that fibre is a bulking agent. Pectin, hemicellulose, and cellulose are examples of fibre. Fibre can be soluble or insoluble. Insoluble fibre is known for softening and bulking stool by absorbing water in the intestines. The risk of developing diverticulosis is reduced, and bowel movement is regularised. Sources of insoluble fibre include potato skins, brans, seeds, brown rice, and vegetables. Soluble fibres aid in reducing the levels of low-density lipoprotein (LDL) cholesterol and postprandial blood glucose and reduce straining with defecation [11].

According to Holesh et al. [11], carbohydrate metabolism starts in the mouth where salivary amylase begins to degrade the sugars. Glucose is one of the final products produced following carbohydrate breakdown by the digestive system. The monomers are now ready for absorption. Below are two major monomers discussed.

It is reported that, in normal human beings, approximately 15–25% of the ingested glucose is metabolised in the liver and the gut. The glucokinase enzyme “activates” glucose by phosphorylation whereby the glucose-carbon-atom on position six links with a phosphate group via its hydroxyl group. This happens in the liver. The glucose-6-phosphate molecule formed undergoes a series of biochemical reactions in a glycolytic pathway to produce two pyruvate molecules. Phosphofructokinase-1 (PFK-1) tightly governs the amount of glucose that undergoes glycolysis. The PFK-1 is inhibited by intracellular excess amounts of ATP (adenosine triphosphate) and citrate. Reports say that the glucose concentration that survives the splanchnic metabolism reaches the systemic circulation. Consequently, a transient increase in the arterial blood glucose level arises from approximately 5 mM/L fasting glucose to 8–10 Mm/L postprandial. Insulin secretion is inevitable therefore, and the arterial glucose is taken up by peripheral organs either independently of insulin (say brain) or under the control of insulin (adipose tissue, skeletal muscle).

Pure fructose ingestion does not trigger insulin secretion or cause markable glycaemia. It is reported that, in case of fructose ingestion, a momentary increment of about 0.5 mM/L in arterial blood glucose takes place. Such a small increment in arterial blood glucose implies that most of glucose is extracted by splanchnic organs. Fructose metabolism takes place mainly in the liver, gut, and kidney. It is reported that, in the aforementioned organs, fructolytic enzymes are present like fructokinase, triokinase, and aldolase B. Fructolysis does not depend on insulin. It is just a biochemical pathway that breaks down fructose to form triose-phosphates viz. dihydroxyacetone phosphate and glyceraldehyde phosphate. Fructokinase and aldolase B are not inhibited by any of the fructolytic products or by signals that arise from cellular energy status [12].

The ingestion of fructose leads to an increment in blood glucose and insulin, compared to an isomolar glucose load. Howbeit, the ingestion of fructose potentiates complete carbohydrate oxidation and energy expenditure in lean healthy volunteers to a larger extent, then in T2DM patients and obese insulin-resistant individuals. In addition, postprandial blood lactic concentrations escalate. The fructolytic pathway converts fructose into lactate and glucose in the splanchnic organs. The glucose produced in the splanchnic organs awaits a secondary oxidation in peripheral tissues. Oral or intravenous fructose boosts glucose synthesis (gluconeogenesis). Surprisingly, glycaemia does not ensue. Also, infusion of gluconeogenic precursors like alanine, lactate, or glycerol leads to gluconeogenesis, but hepatic glucose levels are not affected [12].

### 2.2. Central Nervous System (CNS) and Carbohydrate Metabolism Studies in Relation to T2DM

Defects in insulin secretion cause a metabolic ailment known as diabetes. In addition, insulin resistance is capable of inducing diabetes [13–15]. Hyperglycaemia is a primary indication of diabetes manifestation caused by an abnormal glucose metabolism. A lot of health complications “come along” with diabetes. Type 2 diabetes mellitus (T2DM) affects quality of life and health of patients intensely owing to its high mortality and prevalence. Pathologically and physiologically, the autonomous nervous system (ANS) might take part in nutrient metabolism. Generally, the sympathetic system could potentiate catabolism, while the parasympathetic system could promote anabolism. Evidence is piling up, which support that an escalated sympathetic nervous system activity is associated with pathogenesis of metabolic disorders. Sympathetic denervation improves glucose metabolism and insulin sensitivity; consequently, this implies that the sympathetic nervous system can affect glucose metabolism. When the sympathetic nervous system is activated, acute hyperglycaemia ensues. Such a phenomenon can be prevented by exendin-4. Insulin resistance induced by hypoxia can be relieved by sympathetic nervous system inhibition. Catecholamines mitigate insulin secretion [16, 17].

The prevertebral sympathetic ganglion known as celiac ganglion (CG) and its postganglionic fibres release neurotransmitters like ATP targeting purine receptors [18, 19]. Purine receptors are categorised into two classes, namely P1 and P2. Purinoceptors play a crucial role in the regulation of lipid and glycogen metabolism. In addition to that purinoceptors are involved in the release of insulin [20, 21]. The G-protein-coupled metabolic receptors (P2Y) and the ligand-gated ion channel receptors (P2X) belong to P2 class receptors. The P2Y12 is expressed in both peripheral tissues and central nervous system (CNS). The excitability of sympathetic nerve is controlled by the P2Y12 receptor and is associated with autonomic neuropathy [22]. The receptor might be involved in liver fibrosis, autoimmune pathologies, and platelet aggregation. There is not much information known about the P2Y12 receptor function in nutrient metabolism [16, 23–25].  Table 1 shows P2Y receptor subtypes' distribution, G-proteins, and agonists.

Regulation of nutrient metabolism is carried out by the liver, a key organ. Purinergic signalling controls the pathophysiology and physiology of the liver. The sympathetic CG projects its postganglionic fibres to the liver. In the liver, there is P2Y12 receptor distribution and function [26]. Sympathetic ganglia-P2Y12 receptor is involved in diabetic autonomic neuropathy. The receptor is reported also to be involved in other diabetic disorders [27, 28]. Reduced hepatic glycogenesis, escalated blood glucose, and decreased hepatic glucose uptake may be caused by an excited sympathetic nerve. The function and expression of P2 receptors have been studied in the liver. Nonetheless, it is still ambiguous whether changes in P2Y12 receptor expression have an effect on the CG or liver [16].  Figure 1 shows the purinergic receptors' role in governing the secretion of insulin and the survival of *β*-cells.

Documented reports prove that inflammation plays a key role in the origination and development of a number of metabolic disorders, namely T2DM, obesity, insulin resistance, etc. Neuroinflammation that is related to the autonomic nervous system is capable of contributing to the progression of diabetes. A principal feature of insulin resistance and obesity is presented as a chronic, systemic, low-grade state of inflammation [29, 30]. Activation of inflammasomes is the main molecular mechanism that underlies induction of the inflammatory responses and liver damage under a number of pathological conditions. The pathological conditions include T2DM and development of insulin resistance. There was a suggestion made that inflammasomes link inflammation to insulin resistance [31]. The nod-like receptor protein 3 (NLRP3) inflammasome is a complex that institutes NLRP3, caspase 1, and apoptosis-associated spot-like protein (ASC) [31, 32]. The activation of the NLRP3 inflammasome may lead to cellular inflammatory necrosis and a new kind of a programmed cell death that relies on the activated caspase 1. The above phenomenon is accompanied by the release of proinflammatory factors like interleukin 1-*β* (IL-1*β*). Such proinflammatory factors are known for exaggerating inflammatory response and cell dysfunction [16].

Li et al. [16] carried out research on how the P2Y12 receptor is linked to T2DM. The team made use of short hairpin RNA (shRNA) technology to cut down the P2Y12 receptor in T2DM rats and then probed hepatic glycogen content, inflammatory responses, GK expression, celiac ganglia sympathetic activity, and lipid and glucose profiles. The team noted changes in the hepatic P2Y12 receptor expression and in the celiac ganglia. At the mRNA level, P2Y12 receptor expression was significantly higher in rat livers and celiac ganglia in the T2DM rats than in the control group. The T2DM rats were then injected with the P2Y12 shRNA plasmid, and then a significant decrease in P2Y12 mRNA levels was observed. The results show that shRNA could “undo” the high expression of P2Y12 receptor in T2DM rats. In addition, the team observed that the postganglionic celiac sympathetic nerve discharge of the celiac ganglia markedly increased in the T2DM-rat group compared with the control group. The finding suggests that escalated excitability of the celiac sympathetic nerve is a common phenomenon in T2DM. Nevertheless, treatment with P2Y12 shRNA plasmid normalises the situation. Moreover, principal typical features of metabolic disorders were observed at the early stage of T2DM. Fasting blood glucose (FBG) and fasting plasma insulin (FINS) levels were higher in T2DM rats than in control. In contrast, FINS and FBG levels in T2DM rats treated with the P2Y12 shRNA plasmid were significantly lower. The finding implies that P2Y12 shRNA treatment could normalise changes in FBG and FINS levels and improve insulin resistance in T2DM rats. Furthermore, it was observed that P2Y12 shRNA treatment reduced levels of triglyceride, total cholesterol, and LDL in T2DM rats. A lower hepatic glycogen profile was observed in T2DM rats. Howbeit, upon treatment with the P2Y12 shRNA, the hepatic glycogen significantly increased. A lower hepatic expression of GK mRNA was observed from RT-PCR analysis in the T2DM rats than in the control group. In contrast, hepatic GK mRNA levels in T2DM rats treated with P2Y12 shRNA increased significantly. Western blot results revealed lower GK protein levels in T2DM rats than that in control rats. The GK levels increased upon P2Y12 shRNA treatment. Also, Western blot analysis showed that hepatic NK-*κβ* p65 levels were higher in T2DM rats than in the control group. A markable decease in the hepatic NF-*κβ* p65 levels were noted upon treatment of T2DM rats with the P2Y12 shRNA. Finally, the team examined the effects of P2Y12 shRNA on NLRP3 inflammasome and interleukin-1*β* (IL-1*β*) in T2DM rats. The observation was that, at both mRNA and protein levels, the expression of NLRP3 subunits (ASC, NLRP, and caspase-1) and IL-1*β* was increased substantially in T2DM rats compared with the control group. Notwithstanding, P2Y12 shRNA treatment reversed the escalated levels of NLRP3 and IL-1*β*, exhibiting the beneficial properties of P2Y12 shRNA in playing an inhibitory role of IL-1*β* production and NLRP3 inflammasome.  Figure 2 shows the P2Y12 receptor allows the entrance of a signal from excited CG.

Glucagon is a glucose-elevating hormone that is secreted by pancreatic alpha-cells in the event that blood glucose concentration falls. The hormone then triggers a cascade of biochemical signalling pathways in the hepatocytes that stimulate glucogenesis. The glucose produced then supports the fallen blood glucose level to normalise. Extrinsic electric signals from the parasympathetic and sympathetic ANS also stimulate glucagon secretion. A combination of intrinsic mechanisms, paracrine and juxtacrine, suppress glucagon secretion under normo- and hyperglycaemic conditions. Hypoglycaemia induces glucagon secretion by a mechanism that involves a fall in the ATP/ADP cytosolic ratio and escalated activity of P/Q-type Ca^2+^ channels, causing Ca^2+^ influx. These findings illustrate the crucial vitality of the electrophysiological mechanisms that link glucose metabolism to electrical activity and hormone secretion [33].

Basco et al. [34] conducted an experiment using mice with alpha-cell-specific knockout GK genes. The findings illustrated the crucial role of GK in regulating glucagon secretion from intact islets and *in vivo*. Honzawa et al. [35] came up with a different suggestion concerning glucose-dependent intrinsic mechanism for the control of glucagon secretion. The team mentioned that glucose uptake by sodium-glucose co-transporter 1 (SGLT1) can cause intracellular Na^+^ ion concentrations to be a higher than that of the extracellular compartment. Consequently, secretion of glucagon is triggered. This mechanism is deemed relevant particularly for the paradoxical hypersecretion of glucagon in T2DM. A lot of scientific reports serve as evidence to illustrate that alpha-cells in intact cells are capable of responding to hypoglycaemia by releasing glucagon. In addition, the importance of GK during such phenomena is also documented. Notwithstanding, it is still ambiguous whether alpha-cells are capable of regulating secretion of glucagon intrinsically and whether GK is the glucose sensor linking glucose metabolism to the regulation of glucagon secretion [33].

Moede et al. [33] addressed the above unanswered questions by conducting an experiment where they manipulated GK activity and expression in purified single alpha-cells accompanied with measurements of glucagon release by total internal reflection fluorescence (TIRF) microscopy. In 1996, GK expression in alpha-cells has been done. However, the findings are debatable since the sample that was analysed contained approximately 87% alpha-cells and the rest were other kinds of cells, including beta-cells, which would be suffice to detect GK transcripts. Moede and colleagues managed to obtain 96.6 ± 14% purity of the functional rat alpha-cells. The team examined the hexokinase isoforms that were expressed in rat pancreatic alpha-cells. The results came out as expected: cells that were identified as *β*-cells were positive for GK and negative for hexokinase I, II, and III expression. The most important observation was that all *α*-cells analysed tested positive for GK. Pancreatic alpha-cells were found to express the neuroendocrine GK isoform. Verification of this finding was done by isolating RNA from sorted alpha-cells and performing real-time polymerase chain reaction (RT-PCR) using primers located in the first and seventh exons [36]. The resulted PCR products were subcloned and sequenced. The sequence analysis showed that 60% GK mRNA is encoding the functional B1 neuroendocrine isoform [37]. The rest, that is, 40%, encode neuroendocrine GK nonfunctional variants. Heimberg et al. [38] and Segerstolpe et al. [39] support Moede et al. [33] findings.

The GK enzyme has become a primary target in treating T2DM. Permanent neonatal diabetes mellitus is a severe ailment that occurs as a result of homozygous inactivating mutations in GK. Heterozygous inactivating mutations elevate the threshold for insulin secretion [40, 41]. Glucose kinase regulatory protein (GKRP), as the name says, is a protein that regulates GK in the hepatocytes. The GKRP binds the GK, hence switching off the glycolytic pathway in the event of hypoglycaemia. Many research articles highlight that GKRP mutations that affect its activity, localisation, and expression do not only have impact on glucose homeostasis but also on triglyceride (TG) metabolism [42, 43]. A number of small molecules that serve as GK activators (GKAs) have been found and used in the medical field. Notwithstanding, the activators posed some disadvantageous effects like loss of efficacy over time, increase in TG concentrations, and hypoglycaemia [44, 45]. These effects were linked to ongoing activation of *β*-cells and peradventure related to the development of hepatic steatosis [46–48].  Figure 3 shows glucokinase (GK) phosphorylates glucose during glycolysis.

Patients with GK-activating mutations or GKRP loss-of-function mutations require hepatoselective GKAs that affect neither the GK-GKRP interactions nor GK in *β*-cells. Such “ideal” small-molecule activators can circumvent the adverse effects posed by the GKAs, which have been used in the medical field. Therefore, Vella et al. [48] developed a hepatoselective GKA namely TTP399. The GKA improved glycaemic regulation both in T2DM animal models and patients. Adverse effects like dyslipidaemia, hypoglycaemia, and pathological accumulation of glycogen and TG in the liver were not induced. In addition, TTP339 administration did not seem to perturb GK-GKRP interactions in the presence of normoglycaemia, maybe thus justifying the absence of altered liver function and dyslipidaemia. There was a reduction in hepatic fat in response to TTP399 administration [48].

Hexokinase isoenzyme, known as glucokinase (GK), is expressed specifically in pancreatic islet beta-cells and mature hepatocytes [49, 50]. The GK is a pacemaker enzyme in a glycolytic pathway. It catalyses the first irreversible reaction of glycolysis. The enzyme adds a phosphate group to the carbon atom number six of a glucose molecule, forming glucose-6-phosphate. The product formed can then be metabolised further and stored as glycogen in the liver for future use. GK plays a vital role in regulating glycogenesis and gluconeogenesis in the liver. Therefore, abnormalities in the structure and function of the GK enzyme definitely cause metabolic disorders like T2DM [16].

There is what is referred to as diet-induced diabetes [54, 55]. Scientists have been studying T2DM using high-fat-diet (HFD)-fed mouse models. GK expression in *β*-cells decreased in HFD-induced diabetes according to Lu et al. [27]. Nevertheless, the contribution of decreased GK expression to HFD-induced diabetes is ambiguous. It is reported that HFD-induced defect in *β*-cell function is associated with the downregulation of islet GK. HFD feeding decreases GK mRNA and GK protein by approximately 45%, compared with isoenergetic high-carbohydrate feeding in rats. Previous *ex vivo* studies of islets also showed a decrease in GK mRNA and GK protein following co-culture with palmitic acid [51]. Patients with T2DM were found to have reduced GK expression in the islets [22, 55, 56]. The challenge, however, is that GK is expressed in both hepatocytes and *β*-cells. Therefore, probing the correlation between GK expression and HFD is daunting [57].  Table 2 shows comparison between hexokinase and glucokinase (GK) enzymes.

Regardless of a challenge highlighted above, Lu et al. [57] designed an experiment where they targeted a *β*-cell gene, transferred it into a vector, and then investigated *β*-cell-specific GK expression on *β*-cell function in HFD-induced diabetes. The team made use of the adeno-associated viral (AAV) vector system. The crew observed that overexpression of GK promoted glycolytic flux, activation of ATP-sensitive potassium channel, membrane depolarisation, and an increase in proliferation of Min6 cells. The transduction of *β*-cell GK showed no difference in terms of glucose handling in chow-fed C57BL/6 mice. Adult mice fed with a HFD were found to have reduced islet GK expression, glucose-stimulated insulin secretion (GSIS), and impaired glucose tolerance. Nevertheless, *β*-cell-targeted GK transduction reinstated GSIS and improved glucose tolerance. Perfusion experiments of the islets confirmed restoration of GSIS in isolated HFD islets upon GK gene transduction.

### 2.3. Mechanisms

Based on the studies conducted by Lu et al. [57], restoration of *β*-cell function by *β*-cell-targeted GK overexpression suggests that GK suppression plays an etiological role in *β*-cell dysfunction in HFD-induced diabetes. It is thought that this mechanism is most likely to be regulated through PDX-1, which plays a regulatory role in GK expression [58]. The PDX-1 is downregulated in diabetic victims [59]. A decrease in PDX-1 expression, which leads to reduced GK expression, was observed in rat islets that were incubated in fatty acids. Restoration of GK expression increases glycolytic flux and leads to the induction of glucose response genes like PDX-1 [54, 60, 61]. The mechanism behind increased glycolytic flux by overexpression of the GK is vague. Howbeit, glucose plays a regulatory role in *β*-cell proliferation and GSIS [62, 63]. Overexpression of *β*-cell GK above physiological levels in chow-fed *β*-cells increased glucose utilisation. Glucose induces *β*-cell proliferation via IRS2 and cyclin D2 [64].

According to Vella et al. [48], GK is the target enzyme for T2DM treatment due to the vital role it plays in glucose homeostasis. A number of GKAs have been designed, assessed, and evaluated. At least 30 GKAs are discussed in published preclinical data. GKAs studies in humans and animals showed hypoglycaemia and enhanced *β*-cell function and proliferation. Nonetheless, the clinical trials did not come out well due to adverse effects like hyperlipidaemia, hypoglycaemia, and declining efficacy after prolonged treatment [65]. The proposed mechanism of the above highlighted side effects is that hepatic overexpression escalates hepatic lipogenesis and plasma triglycerides levels in rats [66]. GKAs can be categorised into GKAs that target both the pancreas and liver, hepato-selective GKAs and partial GKAs. Vella and colleagues studied a hepatoselective GKA, TTP399. It is proposed that GK-GKRP interaction is maintained in the presence of TTP399. The TTP399 increased the GK activity in its active conformation. Consequently, TG levels are kept normal. Heavier individuals lost weight upon administration of TTP399. The mechanism underlying this finding requires further studies, including the potential impacts of TTP399 on food intake and appetite.

Reduction in fasting plasma glucagon is a mystery in relation to the study of Vella et al. [48]. Insulin secretion impairment has been the explanation for increased plasma glucagon levels. Notwithstanding, a number of scientists challenged this idea and suggested that insulin signalling impairment explains the elevation of plasma glucagon levels [67]. According to Lee et al. [64], the accumulation of ceramide in *α*-cells of *ob/ob* hyperglycaemic rodents inhibits the suppression of glucagon. The reduction in FBG levels by the TTP399 therapy with no changes in insulin concentrations suggests an improvement in the action of insulin. It is ambiguous if the mechanism highlighted above explains the reduction in fasting glucagon. Needless to say, further studies should be conducted.

According to Li et al. [16], hepatic P2Y12 receptor protein expression was increased in the T2DM rats and the inhibition of the protein (P2Y12) by P2Y12 shRNA caused restoration of glycogen content in the liver. The finding suggests that P2Y12 might be involved in the hepatic dysfunction pathogenesis in diabetic rats. Cell bodies of the sympathetic neurons in the celiac ganglia (CG) project axons to the liver, indicating that the neurotransmission across CG may activate the sympathetic afferents of the liver. The solution, therefore, is the downregulation of the P2Y12 receptor protein expression in both the CG and liver, resulting in the inhibition of the unusual sympathetic excitability, promotion of hepatic glycogenesis, and normalisation of hyperglycaemia. The NLRP3 subunits (ASC, NLRP, and caspase-1) that assemble and activate NLRP3 complex were increased in T2DM rats. This finding is most likely explained by upregulated P2Y12 in the liver of T2DM rats since P2Y12 shRNA mitigated the increments of ASC, active caspase-1, and NLRP. In addition, NF-*κ*B plays a vital role in the inflammatory responses and might be involved in the activation of the NLRP3 inflammasome. Activation of NLRP3 inflammasome complex induces the secretion of IL-1*β*, leading to cell injury and pyroptosis. The P2Y12 shRNA therapy suppressed IL-1*β* release. Therefore, a downgrade of sympathetic purinergic excitability could prevent hepatic inflammation of the T2DM rats, thereby improving dysfunctional metabolism and hepatic insulin resistance [32].

## 3. Conclusions

Type 2 diabetes mellitus (T2DM) is caused by a number of factors namely gene mutations that lead to “underexpression” or overexpression of the GK, GKRP, glucagon, insulin, and PDX-1; *β*-cell dysfunction, hepatic inflammation, unusual excitability of sympathetic nerves, and diet-inducing factors like taking high fat content. Molecular therapy is a promising potent solution to T2DM since the P2Y12 shRNA treatment in T2DM rats mitigated a P2Y12 receptor expression at the mRNA level significantly; increased postganglionic sympathetic nerve discharge (SND); normalised FBG and FINS; improved insulin resistance, triglyceride (TG) levels, total cholesterol (TC) levels, and hepatic glycogen; and reduced NLRP3 complex expression. GKAs are also another good option, particularly hepatoselective GKA like TTP399.

## Figures and Tables

**Figure 1:** The purinergic receptors' role in governing the secretion of insulin and the survival of *β*-cells. The GLUT2 facilitates the entrance of glucose. Glycolysis yields ATP. The ATP produced is used to close up the ATP-sensitive channel, K_ATP_. The K_ATP_ channel is made up of 4 (four) Kir6.2 and SUR1 subunits. When the K_ATP_ closes, the cell membrane potential depolarises and this leads to the opening of the voltage-gated L-type Ca^2+^ channels, generating Ca^2+^ action-potentials. An increase in the cellular Ca^2+^ triggers ATP-insulin-containing secretory vesicles exocytosis. Parasympathetic and sympathetic nerves may also release ATP. Membrane depolarisation and Ca^2+^/Na^+^ influx are facilitated by P2X receptors. P2Y receptors elevate cellular Ca^2+^ and “turn on” protein kinase C (PKC) pathways. Also, other P2Y and adenosine receptors affect the cAMP pathway and possibly Epac signalling. High adenosine concentrations are a “force” that coerces adenosine translocation into the *β*-cell, thus exerting metabolic effects.

**Figure 2:** The P2Y12 receptor allows the entrance of a signal from excited CG. Cleavage of the Casp1 from the NLRP3 leads to cellular inflammatory necrosis. The above phenomenon is accompanied by the release of proinflammatory factors like interleukin 1-*β* (IL-1*β*). Such proinflammatory factors are known for exaggerating inflammatory response and cell dysfunction. The celiac ganglia take part in carbohydrate metabolism, which in turn is linked to neuroinflammation. The P2Y12 shRNA therapy inhibits the excitation of the celiac ganglia, which is associated with overexpression of P2Y12 receptors and then hepatic glucose homeostasis is restored. GLC is glucose, and G6P is glucose-6-phosphate.

**Figure 3:** Glucokinase (GK) phosphorylates glucose during glycolysis. High glucose concentrations cause the release of a bound GK in the nucleus by GKRP. Conversely, high fructose-6-phosphate (F-6-P) concentrations cause GK to be bound in the nucleus by the GKRP.

**Table 1:** P2Y receptor subtypes' distribution, G-proteins, and agonists.

Subtype	Distribution	G-protein	Agonist
P2Y_1_	Broad including skeletal tissue, heart, CNS, platelets	G_q_	ADP
P2Y_2_	Brain, kidney, skeletal muscle, heart, lungs	G_q_	ATP/UTP
P2Y_4_	Vascular smooth muscle, lung, placenta	G_q_	UTP
P2Y_6_	Intestines, spleen, lung, heart, placenta, brain, etc.	G_q_	UDP
P2Y_11_	Dendritic cells, intestine, spleen	G_S_ and G_q_	ATP
P2Y_12_	Hepatocytes, platelets, brain	G_i_	ADP
P2Y_13_	Spleen, brain	G_i_	ADP
P2Y_14_	Haematopoietic cells, intestine, placenta, adipose tissue, heart, brain, etc.	G_i_	UDP/UDP-glucose

**Table 2:** Comparison between hexokinase and glucokinase (GK) enzymes.

Attributes	GK	Hexokinase
Biological importance	Blood glucose homeostasis	Intracellular glucose homeostasis
Clinical significance	Low activity in diabetic patients	Deficiency results in haemolytic anaemia
Inducibility	Determined by the insulin in the liver	Not inducible
Substrate affinity	Lower (K_m_ = 10 Mm/L)	Higher (K_m_ = 0.05 Mm/L)
*V *_max_	Higher	Lower

## Data Availability

The data used to support the findings of this study are included within the article.
